# Artificial Intelligence and Medical Internet of Things Framework for Diagnosis of Coronavirus Suspected Cases

**DOI:** 10.1155/2021/3277988

**Published:** 2021-05-28

**Authors:** Ahmed I. Iskanderani, Ibrahim M. Mehedi, Abdulah Jeza Aljohani, Mohammad Shorfuzzaman, Farzana Akther, Thangam Palaniswamy, Shaikh Abdul Latif, Abdul Latif, Aftab Alam

**Affiliations:** ^1^Department of Electrical and Computer Engineering (ECE), King Abdulaziz University, Jeddah 21589, Saudi Arabia; ^2^Center of Excellence in Intelligent Engineering Systems (CEIES), King Abdulaziz University, Jeddah 21589, Saudi Arabia; ^3^Department of Computer Science, College of Computers and Information Technology, Taif University, Taif, Saudi Arabia; ^4^Aarhus BSS, Aarhus University, Aarhus, Denmark; ^5^Department of Nuclear Engineering, King Abdulaziz University, Jeddah 21589, Saudi Arabia; ^6^Department of Mathematics, King Abdulaziz University, Jeddah 21589, Saudi Arabia; ^7^CIT Department, Faculty of Studies, King Abdulaziz University, Jeddah 21589, Saudi Arabia

## Abstract

The world has been facing the COVID-19 pandemic since December 2019. Timely and efficient diagnosis of COVID-19 suspected patients plays a significant role in medical treatment. The deep transfer learning-based automated COVID-19 diagnosis on chest X-ray is required to counter the COVID-19 outbreak. This work proposes a real-time Internet of Things (IoT) framework for early diagnosis of suspected COVID-19 patients by using ensemble deep transfer learning. The proposed framework offers real-time communication and diagnosis of COVID-19 suspected cases. The proposed IoT framework ensembles four deep learning models such as InceptionResNetV2, ResNet152V2, VGG16, and DenseNet201. The medical sensors are utilized to obtain the chest X-ray modalities and diagnose the infection by using the deep ensemble model stored on the cloud server. The proposed deep ensemble model is compared with six well-known transfer learning models over the chest X-ray dataset. Comparative analysis revealed that the proposed model can help radiologists to efficiently and timely diagnose the COVID-19 suspected patients.

## 1. Introduction

In recent years, Internet of Things (IoT) devices are widely used in a large number of applications such as smart cities, manufacturing, home automation, and medicine [1]. These devices are used to capture information about the physical world through sensors. Nowadays, the healthcare system of the world is overwhelmed due to this COVID-19 pandemic.

There have been more than 21 million confirmed active cases, 55 million recovered cases, and 1.6 million deaths reported in 185 countries as of December 19, 2020. An early diagnosis of coronavirus-infected patients is necessary to stop this outbreak. For this, IoT devices are used for extracting data from COVID-19 patients remotely. This information is transferred to healthcare workers for diagnosis of COVID-19 [2]. These devices not only reduce the burden on healthcare workers but also recognize the unusual patterns from the extracted sensor information. Healthcare workers provide better treatment for coronavirus-infected persons promptly using IoT-enabled devices. There is a need to develop an automatic classification technique by using the information provided by IoT devices. Recently, many researchers have utilized the deep learning models to support various healthcare applications [3].

It is observed from the literature that the chest X-ray modality can be used to classify the subject as COVID-19 (+), pneumonia, tuberculosis, or healthy. It is preferred over other imaging techniques due to cost-effectiveness and having lower risk of radiation exposure to humans.

Figure 1(a) shows the manual chest X-ray modality analysis for the diagnosis of COVID-19 suspected subjects. However, it is a relatively complex and time-consuming task. The radiologists analyzed the white spots, that is, infection in chest X-ray. However, X-ray modalities contain pus and water, which is a challenging and time-consuming process to detect the infection.  Figure 1(b) shows IoT and deep learning-based coronavirus diagnosis framework. The deep ensemble model helps the radiologist to timely diagnose the infected patients.

## 2. Related Work

An IoT-based framework has been designed for early diagnosis of coronavirus-infected patients. Faster region CNN with ResNet101 (FRCR) was utilized to diagnose coronavirus suspected cases. FRCR has achieved an accuracy of 98 % [4]. An attention-based deep 3D multiple instance learning (AD3D-MIL) was proposed for automatic screening of COVID-19 from chest CT images [5]. AD3D-MIL utilized the Bernoulli distribution of labels for efficient learning.

Inspired from the recent success of deep learning models for automated diagnosis of coronavirus, an IoT-based ensemble deep learning framework is designed. The proposed ensemble model will be helpful to the radiologist and medical staff to diagnose the suspected patients as COVID-19 (+), pneumonia, tuberculosis, or healthy. An IoT and deep ensemble model-based framework is designed for the automated diagnosis of COVID-19 suspected subjects. A deep ensemble model is designed such that it ensembles InceptionResNetV2, ResNet152V2, VGG16, and DenseNet201. The medical sensors capture the chest X-ray modalities and diagnose the infection by using the ensemble deep transfer learning model stored in a cloud server. Chest X-ray dataset with four classes (i.e., COVID-19 (+), pneumonia, tuberculosis, or healthy) was used for experimental purposes.

Comparative analysis revealed that the proposed model will be helpful to radiologists for efficiently and timely diagnosing the COVID-19 suspected patients. AD3D-MIL was trained and tested on 460 CT images. A multitask multislice deep learning system (*M*3 Lung-sys) was developed for screening of coronavirus-infected persons using CT images [6].

An auxiliary classifier model was developed to produce synthetic chest X-ray images using the generative adversarial network (GAN). The developed model was named CovidGAN [7]. CovidGAN was used to distinguish COVID-19 from other viral pneumonias. 192 chest X-ray images were used to test CovidGAN. However, the cross-validation is not performed on CovidGAN. Deep learning models were used to detect the COVID-19 suspected cases by using ultrasound, X-ray, and CT scan [8]. VGG19 was utilized to develop an automatic classification technique. The preprocessing technique was used to alleviate the sample bias and enhance the image quality. However, the data fusion techniques can increase the classification accuracy. CNN-based transfer learning framework was proposed for classification of COVID-19 suspected cases [9].

The eight pretrained CNN models, ResNet18, Inceptionv3, SqueezeNet, MobileNetv2, ResNet101, CheXNet, DenseNet201, and VGG19, were used in this proposed framework. This framework was tested on 423 COVID-19, 1485 viral pneumonia, and 1579 normal chest X-ray images. A 3D convolution neural network (3DCNN) was developed to distinguish COVID-19 infection from other infections [10].

DCNN utilized the online attention refinement and dual-sampling strategy. This network was used to extract the infection regions and eliminate the imbalanced distribution of pneumonia-infected regions. DCNN was tested on 2796 CT scan images of 2057 patients. However, the accuracy of the infected area is still not satisfactory. A deep learning-based chest radio classification (DL-CRC) framework was proposed to classify coronavirus-infected persons using chest X-ray [11]. DL-CRC used a generative adversarial network and data augmentation to produce artificial coronavirus infected X-ray images. DL-CRC was tested on four different chest X-ray datasets.

Medical IoT devices have helped a lot to tackle the COVID-19 pandemic. IoT-based deep learning models have been designed to reduce the workload of medical staff and doctors. However, the IoT-based deep learning models that do not consider defensive models against adversarial perturbations remain vulnerable to adversarial attacks [12].

Gianchandani et al. [13] designed an ensemble deep transfer learning model to identify COVID-19 suspected patients. Singh et al. [14] implemented deep neural network-based screening model for COVID-19-infected patients. Singh et al. [15] utilized densely connected convolutional networks to classify COVID-19 patients. Although these models achieve better results, they can be further improved using the ensemble modeling.

From the existing literature, it has been found that the existing models still suffer from the overfitting issue [16, 17]. Ensemble models utilize multiple learning approaches to achieve better classification performance than the individual models [18]. The ensembling of deep learning models yields to significant results when there is a better diversity among the deep learning models. Thus, ensembling is a meta-approach that integrates various deep learning models into one classification model to improve prediction (stacking) or minimize bias (boosting) and variance (bagging).

## 3. Proposed IoT-Based Automated COVID-19 Diagnosis Framework

Figure 2 shows the layer-by-layer architecture of IoT-based automated coronavirus diagnosis framework. It consists of four layers, i.e., perception, network, data storage and processing layer, and application layer. Initially, at the perception layer, medical IoT devices are responsible for collecting various kinds of scans such as X-ray, CT, and ultrasound. Thereafter, these obtained scans are transmitted to the data storage layer with the help of the network (transmission) layer. The network layer may utilize telecommunications, Internet, etc., to transmit the obtained scans.

The data processing/storage layer of IoT network then utilizes deep learning models to classify the subjects as infected or healthy and store the obtained results. Finally, at the application layer, various types of clients such as patients, doctors, or medical staff can utilize the obtained diagnosis results for further treatment or action. The proposed ensemble model for COVID-19 diagnosis is depicted in Figure 3. The proposed model ensembles four well-known transfer learning models such as ResNet152V2 [9], DenseNet201 [9], VGG16 [19], and InceptionResNetV2 [20]. We have used only these models because during experiments on the obtained dataset they achieve good accuracy and have better diversity among the implemented deep learning models.

It has been found that the ensemble of pretrained models provides more efficient results than the individual models. The ensemble technique can extract the optimal features and improve the classification accuracy. Figure 3 shows the proposed ensemble model for COVID-19 diagnosis. 64 neurons are used for the initial dense layer. A fine-tuned transfer learning model is used with many layers to extract the features. To deal with four-class classification problem, the softmax activation function is used. The models are obtained by using epochs = 100 and batch size = 10. During the initial tuning of attributes, fully connected layers with 64 neurons along with dropout of 0.3 and 0.2, respectively, are used to prevent overfitting. Additionally, regularization is also done by considering the concept of early stopping. 0.001 is used as a learning rate.

## 4. Performance Analysis

The proposed DenseNet model is applied to the four-class CXR dataset. The comparison of the proposed ensemble model is drawn with the existing well-known deep transfer learning models. The experiments are performed on a core i7 3.80 GHz, 32 GB RAM, and 15M cache on MATLAB 2020b software. This work uses 20-fold cross-validation to overcome the overfitting problem. 70% of the entire dataset is considered for training purposes.

### 4.1. Dataset

The dataset is collected by incorporating four different existing datasets. The first dataset is obtained from hospitals in São Paulo, Brazil. It consists of 2492 CXR scans that consist of 1262 COVID-19 (+) and 1230 healthy subjects [21]. Additionally, two publicly available tuberculosis datasets of Shenzhen, China, and Montgomery County, USA, are also obtained from the U.S. National Library of Medicine, National Institutes of Health (NIH). The Shenzhen, China's dataset, contains 326 normal and 336 CXR of tuberculosis (+) patients. Montgomery County, USA, has 80 normal and 58 CXR images of tuberculosis (+) patients. In total, 1663 COVID-19 (+) patients, 401 pneumonia subjects (viral as well as bacterial pneumonia), 394 tuberculosis patients, and 2039 images of healthy persons are used for experimentation. Data augmented are also implemented using random rotation, random cropping, and random blurring.

### 4.2. Comparative Analysis

Figure 4 shows the training and validation analysis of the proposed model. It clearly shows that the proposed model achieves better training and validation results and is not much affected by overfitting issues.

Figure 5 shows the confusion matrix analysis of the proposed ensemble model on the testing dataset. For COVID-19 class, the overall accuracy is 99.6%. For healthy patients, the proposed deep ensemble model shows an accuracy of 99.2%. For pneumonia class, the overall accuracy of the proposed deep ensemble model is 99.4%. The tuberculosis class has received an accuracy of 99.1%. The proposed model achieves the excellent overall classification with an overall accuracy of 99.3%. Thus, the proposed model is not much affected by the overfitting problem.

Table 1 depicts the validation analysis of the proposed model. The results reveal that the proposed framework provides better results than the existing deep learning models. The proposed framework achieves better performance than the existing models in terms of accuracy, *F*-measure, sensitivity, specificity, and area under the curve (AUC) by 1.2832%, 1.1837%, 1.3281%, 1.3928%, and 1.2837%, respectively.

### 4.3. Discussion

FRCR has shown an accuracy of 98% on chest X-ray images. DL-CRC achieved the classification accuracy of 93.94%. The sensitivity, specificity, and accuracy obtained from 3DCNN were 86.9%, 90.1%, and 87.5%, respectively. The classification accuracy, specificity, and sensitivity achieved by CheXNet were 97.9%, 97.9%, and 98.8%, respectively. VGG19 achieved an overall sensitivity of 93%. The classification accuracy obtained from CovidGAN was 95%. The classification accuracy obtained from ACCA was 91.1%. AD3D-MIL attained the classification accuracy of 97.9%, AUC of 99%, and kappa score of 95.7%. Therefore, the proposed approach outperforms these techniques with an accuracy of 99.2 and *F*-measure of 99.17. Additionally, the proposed ensemble model achieves sensitivity, specificity, and AUC as 99.12, 99.07, and 99.21, respectively. Thus, the proposed model is more reliable in terms of performance compared to the existing COVID-19 diagnosis models.

## 5. Summary and Future Directions

The paper offers a real-time communication and diagnosis of COVID-19 suspected cases. An IoT-based automated coronavirus diagnosis framework was designed by using the ensemble deep learning. The proposed framework has ensembled four deep learning models such as ResNet152V2, InceptionResNetV2, VGG16, and DenseNet201. The performance of the proposed model was implemented on four-class chest X-ray datasets. Comparative analysis has shown that the proposed model can help radiologists to efficiently and timely diagnose the COVID-19 suspected patients. The proposed framework achieves better performance than the existing models in terms of accuracy, *F*-measure, sensitivity, specificity, and area under the curve (AUC) by 1.2832%, 1.1837%, 1.3281%, 1.3928%, and 1.2837%, respectively.

The hyperparameter tuning issues of deep transfer learning models remain to be addressed. An efficient hyperparameter tuning can enhance the results of the deep transfer learning models. Moreover, it will be important to extend the proposed model to diagnose chest CT and ultrasound images. Additionally, the proposed model can be used for other fields to build a multidisease classification model.

## Figures and Tables

**Figure 1:** COVID-19 diagnosis models: (a) manual COVID-19 diagnosis model and (b) IoT-based automated COVID-19 diagnosis model.

**Figure 2:** Layer-by-layer architecture of the proposed IoT-based automated COVID-19 diagnosis framework.

**Figure 3:** Proposed ensemble deep learning model.

**Figure 4:** Training and validation loss analysis.

**Figure 5:** Proposed ensemble deep learning model confusion matrix analysis of the proposed ensemble model on testing dataset.

**Table 1:** Comparative analysis of the proposed ensemble framework and the competitive deep learning models.

Model	Accuracy	*F*-measure	Sensitivity	Specificity	AUC
CNN	97.32 ± 0.92	97.95 ± 1.21	98.02 ± 1.18	98.18 ± 1.17	97.97 ± 1.03
VGG16	98.12 ± 1.06	98.19 ± 0.95	98.02 ± 1.18	98.19 ± 1.18	98.08 ± 1.21
ResNetV2	98.31 ± 0.98	98.51 ± 1.08	98.21 ± 1.04	98.20 ± 0.94	98.16 ± 0.94
DenseNet201	98.82 ± 0.92	98.73 ± 0.92	98.72 ± 0.79	98.42 ± 1.04	98.48 ± 0.89
Inception V4 network	98.73 ± 0.96	98.83 ± 0.83	98.63 ± 1.05	98.42 ± 1.12	98.62 ± 0.91
ResNet152V2	98.82 ± 0.82	98.82 ± 0.58	98.74 ± 0.83	98.83 ± 0.85	98.85 ± 0.79
Proposed model	99.2 ± 0.58	99.17 ± 0.61	99.12 ± 0.72	99.07 ± 0.79	99.21 ± 0.67

## Data Availability

No data were used to support this study.
